# COVID-19 as an “Infodemic” in Public Health: Critical Role of the Social Media

This article has been retracted.

**DOI:** 10.3389/fpubh.2021.610623

**Published:** 2021-03-18

**Authors:** Debanjan Banerjee, K. S. Meena

**Affiliations:** ^1^Department of Psychiatry, National Institute of Mental Health and Neurosciences, Bengaluru, India; ^2^Department of Mental Health Education, National Institute of Mental Health and Neurosciences, Bengaluru, India

**Keywords:** COVID-19, coronavirus, pandemic, misinformation, social media, infodemic

## Abstract

The Coronavirus disease 2019 (COVID-19) pandemic has emerged as a significant and global public health crisis. Besides the rising number of cases and fatalities, the outbreak has also affected economies, employment and policies alike. As billions are being isolated at their homes to contain the infection, the uncertainty gives rise to mass hysteria and panic. Amidst this, there has been a hidden epidemic of “information” that makes COVID-19 stand out as a “digital infodemic” from the earlier outbreaks. Repeated and detailed content about the virus, geographical statistics, and multiple sources of information can all lead to chronic stress and confusion at times of crisis. Added to this is the plethora of misinformation, rumor and conspiracy theories circulating every day. With increased digitalization, media penetration has increased with a more significant number of people aiding in the “information pollution.” In this article, we glance at the unique evolution of COVID-19 as an “infodemic” in the hands of social media and the impact it had on its spread and public reaction. We then look at the ways forward in which the role of social media (as well as other digital platforms) can be integrated into social and public health, for a better symbiosis, “digital balance” and pandemic preparedness for the ongoing crisis and the future.

## Coronavirus Disease 2019 (COVID-19): The Global Problem Statement

The coronavirus disease 2019 (COVID-19) caused by Severe Acute Respiratory Syndrome (SARS)-Cov-2 virus, emerged into a pandemic within a month of its emergence. On January 30th, World Health Organization (WHO) declared it a “public health emergency of international concern” and termed it as the “worst pandemic” the world has seen so far since the Spanish Flu of 1918 (1). The virus though less fatal is much more contagious than its early congeners causing SARS and Middle East Respiratory Syndrome (MERS) with the faster human-human transmission, already affecting more than 109 million globally, the numbers rising as we speak (World Health Organization, as of February 15, 2021). As economies have slashed, travel restrictions imposed, and international borders sealed, billions stay quarantined at their homes as a strategic measure of social distancing used to contain the outbreak. The uncertainty of a pandemic and chronic isolation can lead to panic and psychological distress, which gets further worsened by the plethora of information pumped into the masses every day, predominantly by social media (2). The isolation and anxiety lead to increased media penetration in various nations, further snowballing the effects. In an online survey done on 1,310 people in Italy, digital media usage had increased during the lockdown, with sleep-wake cycle disruptions and lowered sleep quality (3). The authors highlighted the need for interventions to prevent this social disruption by increased media usage that can potentially contribute to the falsification of information. Another internet-based study assessing the relationship between media use and acute psychological outcomes in China reported media engagement to be associated with more negative affect, anxiety, stress and sleep disturbances (4). The average use of digital media among the participants was also reportedly increased. Worsening of sleep quality and quality of life have been reported in other studies (5).

COVID-19 has been referred to as a “digital pandemic” due to the multitude of information in various forms that have been circulated since it got first detected in Wuhan, China. As the case numbers increased, the shared information rose exponentially due to all the social media platforms competing in their speed, coverage, and penetration (6). Given that more than three billion individuals use social media regularly, and for prolonged periods, it becomes the primary source of information and communication, especially during a crisis, irrespective of the authenticity of the sources (7). Out of this bulk of facts processed regularly, a substantial proportion is either myth, rumors, pseudoscience or altered facts: contributing to misinformation. Based on health-risk perception theory, the fear of an “unknown” illness without a definitive cure creates uncertainty, leading to anxiety and increased sharing of misinformation, unaware of the sources (8). COVID-19 risk perception has been shown to significantly affect socioeconomics and media attention in various countries (9, 10). Thus, it can be hypothesized that any senseless forward of a message, meme or video can snowball the effect, if in wrong hands. Termed as “misinfodemic”, this epidemic of “shared misinformation” has become rampant during this pandemic, spreading faster than the virus itself (11). A global analysis of Google Web Searches and Instagram Hashtags showed that countries with a higher number of COVID-19 cases had a higher number of related Google queries (12). “Coronavirus ozone”, “coronavirus laboratory”, “coronavirus 5G” and “coronavirus conspiracy” were widely being circulated on the web. More than two-thirds of Instagram users used the hashtags “COVID-19” and “coronavirus” to share virus-related information, which suggested the growing interest in infodemic monikers and need to be vigilant about the same. Similar findings were also reported by network analysis of “medical news frames and conversations” on Twitter from South Korea (13). Tweets containing “coronavirus” had faster communication and spread, while medically framed news articles containing information about COVID-19 were perceived to be more popular.

Isolation and anxiety further increase the “digital screen time” and the continued “information overload” can have dire public health consequences (14). Increased information consumption can have a significant and long-lasting impact on social behavior, which assumes utmost importance in biological disasters such as pandemics. How can we contextualize this “misinformation”? Scheufele and Krause (15) reported that it could be defined in various ways. The operational definitions do not differentiate between “incorrect information” and disinformation. In the context of COVID-19, Krause et al. (16) broadly defined misinformation as “any message that conflict with the best available evidence related to the pandemic, and that would likely not be corrected if it was challenged.” In this article, we briefly highlight the impact of such misinformation concerning COVID-19, the factors enhancing its spread, and how social media could be used more efficiently at times of such crisis.

## COVID-19 As an “Infodemic” in Public Health: The Impact

Compared to the earlier outbreaks of SARS, MERS, influenza and Ebola, the “digital consumption” of facts and statistics have been much more during this time (17). There has not been a day since the advent of COVID-19 that memes, videos, audio clips, text messages, or even treatment charts have not been circulated on social media. They range from conspiracy theories about the origin of the novel coronavirus and “patient zero” to homemade remedies like tea and garlic that can cure COVID-19. The impact of information is directly related to the usage of social media. This article, however, mentions that contrary to the prevalent, popular belief, COVID-19 is not the first “digital infodemic” of the modern world. In the recent past, the outbreaks of Influenza, Zika, and Nipah viruses had caused rapid dissemination of information through social media that contributed to public behavior in terms of panic, health care, and precautionary measures (17).

However, since the first case of COVID-19 struck the world, the detailed worldwide data as that of the respective geographical distributions, are being consistently fed to the masses with consumption increasing compulsively. Even factual information is updated every minute on various platforms, including numbers of cases and deaths with zonal and geographical distributions. Statistics, graphs, and figures presented to us every day have hijacked the daily conversation and communication. It is a well-researched fact that during any public health crisis, there is an immense and immediate need for credible information and effective crisis communication (18). The spread of information or misinformation in the target audience has already had a critical impact on the understanding and interpreting the outbreak in countries like Italy, Spain, and the United States (19). In a nationally-representative study, 47% of Americans were exposed to the news that COVID-19 was “completely made up” (20). An earlier study from the same group showed that misinformation could affect public health in the same way as it affects “terrorism, immigration, sexism and racism” in the country (21).

The commonly prevalent myths are the virus being dormant in throats that is amenable to hot water gargling, the use of tea and garlic for killing the virus, using magico-religious practices, using breathing exercises to cleanse the respiratory airway of the virus, etc. (17). Irrespective of the origin, these get spread to every other part of the world *via* social media. Certain times these are claimed to be from authentic sources like WHO, Centre for Disease Control and Prevention (CDC), etc. without sufficient evidence. The “false” association of these prominent public health agencies with fake news increases the perceived credibility, consumption and consequently the spread. Also, facts like COVID-19 being used as a biological weapon and permanence of viruses in the air for more than a month have added to mass hysteria and political tensions^1^. In the recent past, it has added to the mutual blame, othering, and prejudice against particular nations, as being responsible for the spread of the virus (22). Internally in countries, the association of this infection with hygiene and sanitary measures has generated stigma and marginalization against migrants, daily laborers and homeless individuals in European countries, the United States, and South Asian countries like India and Bangladesh (23). An infoepidemiology study by Hu et al. (24) showed that people used stigmatizing terms like “Wuhan pneumonia,” “Wuhan coronavirus,” “Chinese virus,” etc. in Google Search with high collective heterogeneity of crowd behavior, rather than the official terms. The unintended effects have been perceived stigma toward the Chinese communities and those who physically resemble them in other nations. In another infodemiology study on social media data by Liao et al. (25), the content patterns identified in personal and government posts were related to knowledge about the infection, guidelines and administrative policies. As the pandemic evolved, individual posts showed decreased empathy and increased attribution of blame toward other individuals. The authors suggested the importance of closely monitoring social media content during such outbreaks. Yet another study evaluated the quality and readability of online information related to COVID-19 by critically analyzing 110 websites using the Health on the Net Foundation Code of Conduct (HONcode), the Journal of the American Medical Association (JAMA) benchmark, the DISCERN instrument and Google ranking (26). While only 1.8% of the websites had the HONcode seal, 10% of them had all the four necessary criteria as per JAMA. Based on the DISCERN score, none of the websites had a high score, whereas 70% of them scored in the “low” category. The authors implied that most of the misinformation related to the outbreak is obtained from the media, and the spread is much faster compared to non-COVID content.

Besides social stigma, the generated misinformation can also lead to adverse health consequences. A vulnerable mind accepts any easy solution, and that leads to faulty treatments, unnecessary hoarding of medications, and protective equipment, as well as chaos, which can have adverse psychosocial consequences. An example of this is people stocking up antivirals like ritonavir and lopinavir and antimalarials like hydroxychloroquine (HCQ), the moment these medicines appeared on the news. This has led to a shortage of medication supplies for their intended uses and increasing cardiotoxicity due to self-medication of HCQ^2^. The selective appearance of HCQ on the media as a “life-saving” drug against COVID-19 has overshadowed the strictly prescribed guidelines for its use, and the weak scientific evidence for its widespread use against the coronavirus (27). A cross-country comparison of public awareness, rumors and behavioral responses to the pandemic in 12 nations using internet surveillance data showed “windows of missed opportunities” in most countries to increase public awareness when the caseloads were low (28). Rumors and misinformation were responsible for a surge in herbal remedies in China and antimalarials globally as perceived “cures” for COVID-19. The study further revealed that timely fact-checking of such fake news helped in mitigating panic buying of these non-evidence-based remedies. Such a selective portrayal of scientific literature generalizing the effects of treatment in its early phases, especially during a crisis like pandemics, can quickly generate a “false hope” with overuse against the recommended safety guidelines.

Curiosity is the basic human instinct, and socialization increases it. Incomplete understanding, partial or biased interpretation, hearsay, rumor-mongering and inadequate communication are the main ways that give rise to health-related misinformation (29). Qualitative studies on social media and human behavior during the earlier outbreaks of SARS and Influenza have revealed that false but commonly held beliefs, generalization of traditional beliefs, the theory of negativity bias, social modeling of rumors, over-analysis and faulty interpretation of science (pseudo-science), motivated and fear reasoning as well as the amplification effect of media as potential mechanisms for infodemic spread (29, 30). Banerjee and Rao (30) while discussing the psychology of misinformation during the pandemic, highlights social learning, attributional bias and various other cognitive biases for the potential spread of fake news. Social media is portrayed as a “double-edged” sword with the potential to trigger disinformation, social stigma and “othering” and be used for fact-checking, public awareness, health surveillance and health education. The authors refer to a healthy “digital balance” integrating public health and technology for effective health communication during the pandemic. The penetration of social media has undoubtedly increased over recent years, that is what probably makes COVID-19 different and socially more alarming than many other fatal epidemics that occurred earlier like the Spanish flu and cholera, where communication was highly restricted to certain pockets in the absence of such widespread penetration of social media (23). Croucher et al. (31) reported increased xenophobic sentiments, social stigma, racism and prejudice against the “Asian” communities in the United States (U.S.) due to increased use of social media during the pandemic. The results revealed that participants tend to believe the “facts” shared on social media as “truths,” gender differences in the type of prejudice (intergroup anxiety for men and a symbolic threat for women), and enhanced chances of viewing the “Chinese” as a threat in those with increased usage of social media.

## Integrating Social Media for Pandemic Response: A “Double-Edged” Path

Is information dissemination then all that bad? Definitely not. In modern days of digitalization, data and management protocols reach corners of the world in a blink leading to mutual learning and shape research so that humankind can stand united against this dreadful disease. Social media shares a crucial role here. The optimal harnessing of this digital tool for trustworthy information, emotional preparedness, and community resilience during a pandemic can help contain the outbreak (32). Especially when there are worldwide shutdown and mass-isolation, social media can provide constructive information, help relieve loneliness, and fight misinformation. Integrating social media tools to generate language and community congruent infographics have been used during the first wave of COVID-19 infection at Wuhan, with rapid dissemination among the health-care workers and general masses (33). Studies conducted on the Knowledge-Attitude-Practice (KAP) gap survey showed an enhanced understanding of the illness, improved knowledge of precautionary measures, reduced panic and better communication of information (33). As the use of platforms like Whatsapp, Facebook, and Instagram is rapidly increasing, especially in adolescents, they can be potentially useful targets for community sharing of knowledge related to pandemics. A similar use of social media has been used for integrating primary, secondary, and tertiary levels of health care during the Zika outbreak in China and the Ebola outbreak in Africa (34). These studies show that if social media can be channelized for information sharing, the reach is speedy, and effects are significant, helping fight an outbreak, where “time” is the key. Controlling the compulsive use, identifying the vectors of misinformation, and educating the differentiation of “true-fake” news were the notable challenges.

Larger social media teams are gradually getting involved in fact-checking and debunking fake news. They have got linked to reliable sources like WHO, CDC, and the National Institute of Health (NIH). Facebook, through the news feed, Twitter, and other social media sites, are directing people who are searching for coronavirus related data to Google scholar and Pubmed, which can then pull out relevant scientific articles. The content of search is recorded to refine searches later on, and search data is pooled to study the common sources of misinformation and false facts (35). Awofeso (36) has suggested “re-inventing” social media platforms as trustworthy learning and health-communication tools. This will necessitate the involvement of all stakeholders such as regulation and monitoring of misleading content, self-regulation of influential persons with regards to their pandemic-related statements and reactions on social media, as well as ensuring widespread digital health literacy tailored to the “need for information” about the outbreak (36). This helps to identify “vectors” of misinformation, which are commonly the sources or “identifiers” of information spread (e.g., a particular piece of news on the use of garlic having antiviral effects in throat being generalized for COVID-19 and this article being circulated as evidence to substantiate the false claim). Fact-checking has been reported as an effective form of health-risk communication during the pandemic (16). Misinformation is in itself considered to be a “meta-risk” to public health by interacting and compounding public's perceptions of the facts, especially during a global-scale outbreak like COVID-19 (16). However, the focus needs to be beyond just fact-checking. Fact-checking responses as risk-communication though necessary, are on their own insufficient to counter misinformation (11). As mentioned before, the multiple other factors like social stigma, panic, fear of infection, cognitive biases, racism, xenophobia and international tensions, that contribute to the propagation of “fake news” need addressal. Highlighting the motives behind disinformation, public awareness through collaborative action between media, health professionals and administration, as well as “authentication” of social media content and accounts have been proposed as other strategies during the pandemic besides fact-checking (11).

The various ways in which social media can be used during pandemics, such as COVID-19 to achieve a “digital balance” in public health are proposed in Table 1 (30).

**Table 1:** Possible roles of social media during pandemics.

**Role of the social media during pandemics**	**Processes involved**
Fighting false news and misinformation	• Using diagnostic and referral health tool (Example: Facebook Preventive Health tool) • Individualized approach for evaluation, testing, counseling based on reported symptoms • Highlighting and debunking rumors, providing relevant data • Integrating data from search engines (like Google QHub) to understand and study trends of misinformation • Prevent information-overload and content related to xenophobia, stigma and prejudice
Enabling digital health literacy	• Video-conferences and webinars • Live platforms (like Facebook, Instagram) for awareness campaigns • Liaison between journalists and physicians
Helping research during crisis	• Search data can be pooled and studied to understand the unmet needs • Community public health research
Resource and psychological preparedness during pandemics	• Liaising with public health platforms (WHO, CDC, ICMR, etc.) and forums like “worldometer” to update statistics and trends of ongoing infection • Integrating essential service location and contact tracing using special applications • Counseling, mental health crisis intervention and suicide prevention
Crisis communication	• Identifying priorities, providing relevant facts and precautionary measures
Fighting stigma	• Assisting community awareness campaigns through advertisements and promotion • Incorporating popular/public figures in the media • Information-Education-Communication (IEC) activities • Socio-culturally and linguistically sensitive infographics
Facilitating public health needs	• Geo-location facilities for identifying hotspot zones and case loads • “COVID-free” content for recreational purpose • Special services for those in quarantine • Training and health-communication between tertiary and primary health care
Addressing mental health	• Social connectedness in community and enhancing mutual support • Mitigating loneliness • Increasing “COVID-free” content to reduce panic • Fostering optimism and hope • Humanizing mental illness • Providing authentic information of mental disorders and treatment • Advocating and promoting mental wellbeing through media programs (especially for the vulnerable groups and those with pre-existing psychiatric disorders) • Counseling using cyberspace • Sensitive reporting of suicides (including celebrity suicides)
Aiding healthy use of media	• Advocate healthy use of technology • Regulated timelines and content

*WHO, World Health Organization; CDC, Center for Disease Control and Prevention; ICMR, Indian Council of Medical Research*.

## The Way Forward: Role of “Digital Health Literacy”

The need for a comprehensive health education program to address COVID-19 has been mentioned by the WHO in its Situation Reports (1). Health Literacy in any community evolves out of understanding our health, which in turn aids us to become responsible individuals to lead an optimally healthy life. The lacunae of health literacy among the public increase stigma and myths and misconceptions related to COVID-19 (37). Hence, stigma gets all the more strengthened due to lack of proper education methods and improper information dissemination. Proper information sharing and health communication through mass media among the community can aid in health literacy. The deep-rooted stigma, lack of support and the ignorance, rapid news of fake information spread on social media platforms and devices being some of the factors among the community has made it crucial to assess the level of health literacy of the public so that proper steps can be taken to increase accurate information on COVID-19 for better treatment-seeking (37). It is also vital to understand that the impact and snowballing of “false news” related to “attractive and easy cures” are much higher than accurate news. As mentioned before, the troubled human mind often resorts to believing the “psychologically expected fact” irrespective of logical reasoning and hence the societal spread is enhanced (38). By the time, a certain “false news” is debunked on a particular platform, and the originally generated false news has probably already spread among millions, many of whom either might not come across or believe the fact. Such credibility generating information also needs an active collaboration between the media and scientific professionals (experts in the respective fields of public health, infectious diseases, and epidemiology), with the training of the primary health care workers in identifying and debunking misinformation as well as helping the community with simple and relevant sources of updated information (38). A psychosocial community-based toolkit for COVID-19 proposed by Banerjee and Nair (39) based on the Zikavirus model also incorporates the integration of media, influential social figures and primary healthcare workers into the public health framework for better preparedness during the pandemic.

Besides, care needs to be taken to look into culturally specific mediums of communications as they are critical in conveying information in certain communities. The critical adverse effect of low health literacy could also be that of infiltration of news related to demand and shortage for essentials at hospital settings, widespread news of non-scientifically tested treatments for curing, myths and misconceptions, and widespread discrimination. The use of various audiovisual and print mediums can help in proper information dissemination as they can reach out to a large number of people in no time. Sharing the success stories of people suffering from COVID-19, higher recovery rate, decreased mortality rate can encourage the communities to look at it positively. People working in the print and electronic media need to work ethically and responsibly in providing credible and authentic sources of information related to COVID-19. The inclusion of a comprehensive health education program with a focus on developing multiple methodologies in disseminating information on COVID-19 by the government for proper awareness will not only help the health and frontline workers but also, in turn, increase the health literacy among people in the community at large (40). These can achieve by developing various IEC [Information Education Communication] resources like brochures, videos, infographics, various digital platforms, podcasts, campaigns (print and online) blogs, vlogs and various other social media platforms. Overlooking the limitations, social media can play a critical role in disseminating information in addressing the pandemic. This integrative role can thus help the psycho-social and public health at large.

We propose the following ways in which media and technology can be used at times of pandemics to aid public and social health. Some of these pertain exclusively to social media, while others involve the use of digital platforms.

### Debunking Misinformation

To understand the origins and spread of misinformation, coordinated efforts to identify and disrupt its sources and prevent its circulation are need of the hour. Social media-based diagnostic and referral health tools (Example: the Facebook Preventive Health tool, Twitter geo-detector) can be used to adopt an individualized approach to COVID-19 cases directing them to appropriate sources of evaluation, testing, and management based on their reported symptoms. A study in Jordan sampled 2,555 social media users *via* web-questionnaires and reported healthy use of social media platforms to have a significant positive influence on public health protection, which in turn was mediated by public health awareness and public health behavioral changes (41). Studies have also reported using health surveillance systems in effective fight against infectious disease outbreaks (42). A similar approach has been used before for cardio-vascular risk and cancer screening.

### Psychological Help and Establishing Crisis-Communication

To raise awareness, help mobilize the vulnerable population like the elderly, and guide the helping agencies to the socially disadvantaged population: psychological first aid services can be provided by artificial intelligence or even counseling services incorporated as per need within the social media networks. They are surely not the replacement for mental health professionals but can help build community resilience during the current crisis.

### Facilitate Digital Learning

When social distancing has impaired group discussion, webinars and videoconferences can be ideal for sharing knowledge and information between public health experts about treatment and prevention of COVID-19; similar networks can be used to facilitate collaboration between the media and physicians to debunk health-related misinformation. Live social media platforms can carry out these useful awareness programs to the masses, also helping them get their queries addressed.

### Pandemic Preparedness

Social media can form the backbone of the public health system, and lessons learned from COVID-19 can help prepare for futuristic infectious threats. When the first case gets detected globally, the upcoming trends of the outbreak can be monitored in a systematic and regulated way, rather than generating panic with false messages.

### Aiding Scientific Research

The immense amount of search results can be pooled and harnessed for understanding the transmission and trajectory of a pandemic. Electronic medical health records can be tallied with reported symptoms to gauge the personalized risk for individuals. Throughout COVID-19, this data can be used for systematic research by the scientific and media communities.

### Handling Stigma

Social media pages/posts have become an easy tool for people to spread hate and racism among certain people, races, communities, and places. Anti-stigma measures like positive message campaigns, development of IEC material, print and audio-visual aids can play a pivotal role in reducing stigma. People tend to use this more during the current situation, which can improve the recognition of mental and social health. Such habits developed now can outlast the pandemic for the better.

### Promoting Public and Mental Health Needs

Especially during the worldwide isolation and quarantine, social media use has served both as an informative and recreational tool for the masses. “COVID-free” content needs to be incorporated into the updates, related to other information or entertainment. Brief messages or infographics can promote the essential precautionary measures and need for psycho-social well-being, which will be more useful than the bulk of epidemiological numbers, that can further arouse panic. Such strategies have been part of earlier community-campaigns during the SARS and Zika outbreak, which has improved the overall satisfaction of social media usage and quality of life (43).

### Awareness Through Social Media About Its Regulated Use

Media platforms can be used for awareness against its compulsive use. Regulated timelines are better sorted out with the help of administrative policymaking. Unnecessary forwards and spreading misinformation need to be prohibited. The adverse effects of social media use can be propagated on the same medium itself. That becomes more acceptable to the public.

## Conclusion

WHO has identified COVID-19 as one of the greatest threats to public health, and the public response has been affected by a global infodemic (or misinfodemic), like never before (35)! This is probably a price we pay for globalization. Over-abundance of information can cause information pollution, where it becomes difficult to tease out “what is authentic” at times of crisis, without reliable sources. The various online media platforms may rush to publish a piece of information without verifying as it is a global challenge to report facts when they are changing every hour. Certain vulnerable communities like the children, adolescents and older adults need to be specially protected from the effects of misinformation and digital health literacy can be promoted and advocated by the social media. History has taught us that at times of biological disasters, social media penetration is high, and it can have a marked impact on the public response. Apart from misinformation contributing to mass-hysteria and panic, faulty treatments, competitive health care, and non-compliance to precautionary measures are among the other burdens of public health. Simultaneously, various community programs during pandemics have tried to borrow from social media in disseminating useful information for community awareness, treatment collaboration and research, which eventually help in fighting the outbreaks. Overall, social media is a double-edged sword. The lessons learnt throughout this COVID-19 pandemic can help make public health and social media more symbiotic and mutually stronger. This integrative role of social media in public health promotion can help facilitate better psycho-social and global well-being.

## Author Contributions

All authors were involved in conceptualization, literature review and drafting the manuscript. The final version was read and approved by all authors.

## Conflict of Interest

The authors declare that the research was conducted in the absence of any commercial or financial relationships that could be construed as a potential conflict of interest.

## Footnotes

^1^BBC. May 4th, 2020. https://www.bbc.com/news/av/technology-52477361 (accessed on February 15, 2021).

^2^https://www.bloomberg.com/news/articles/2020-03-20/hospitals-stockpile-malaria-drug-trump-says-could-treat-covid-19 (accessed on April 7, 2020).
